RETRACTED

# miR‐664a‐3p functions as an oncogene by targeting Hippo pathway in the development of gastric cancer

**DOI:** 10.1111/cpr.12567

**Published:** 2019-03-18

**Authors:** Lu Wang, Bowen Li, Lu Zhang, Qing Li, Zhongyuan He, Xuan Zhang, Xiaoxu Huang, Zhipeng Xu, Yiwen Xia, Qiang Zhang, Qiang Li, Jianghao Xu, Guangli Sun, Zekuan Xu

**Affiliations:** ^1^ Department of General Surgery The First Affiliated Hospital of Nanjing Medical University Nanjing China; ^2^ School of Medicine Southeast University Nanjing China; ^3^ Jiangsu Key Lab of Cancer Biomarkers, Prevention and Treatment, Jiangsu Collaborative Innovation Center For Cancer Personalized Medicine, School of Public Health Nanjing Medical University Nanjing China

**Keywords:** GC, Hippo, metastasis, miR‐664a‐3p, MOB1A, proliferation

## Abstract

**Objectives:**

It has been accounted that miR‐664a‐3p has different functions in several malignancies; however, the precise role and underlying mechanism in gastric cancer have not been elucidated. Our study aims to explore the function of miR‐664a‐3p on the progression of gastric cancer (GC).

**Methods:**

qRT‐PCR was applied to detect the expression of miR‐664a‐3p in GC tissues and cells. The functions of miR‐664a‐3p on GC in vitro were examined by cell proliferation assay, and transwell assay. Related proteins of epithelial‐mesenchymal transition (EMT) and signal pathway were evaluated by Western blot and immunofluorescence analysis. The bioinformatic, dual‐luciferase assay or ChIP assay were employed to identify the interaction between miR‐664a‐3p and its target gene or Foxp3. The effects in vivo were investigated through a mouse tumorigenicity model.

**Results:**

miR‐664a‐3p was frequently upregulated in GC tissues and cells. Elevated expression of miR‐664a‐3p significantly promoted proliferation and invasion in vitro and in vivo. MOB1A was confirmed to be a target of miR‐664a‐3p and restoration of MOB1A attenuated the effects of miR‐664a‐3p. A series of investigations indicated that miR‐664a‐3p contributed to EMT process and inactivated the Hippo pathway by downregulating MOB1A.

**Conclusion:**

Taken together, we revealed that miR‐664a‐3p functions as an oncogene by targeting Hippo pathway in the development of gastric cancer.

**Abbreviations**
EMT: epithelial‐mesenchymal transition
Foxp3: forkhead box protein 3
GC: gastric cancer
LATS2: large tumour suppressor 2
miRNA: microRNA
MOB1A: Mps One Binder Kinase Activator 1A
PBS: phosphate‐buffered solution
TAZ: transcription co‐activator with PDZ‐binding motif
YAP: Yes‐associated protein

## 1 INTRODUCTION

Gastric cancer (GC) remains the second leading cause of cancer‐related mortality worldwide, although the incidence has reduced over past six decades.^1^ Currently, GC is generally diagnosed at an advanced stage with the development of diagnosis technology.^2^ Despite the improvement in the treatment of GC, including radical resection, chemotherapy, radiotherapy and molecular targeted therapy, the 5‐year survival rate of patients with advanced GC is only 5%‐20%.^3^ The poor clinical outcomes of advanced GC patients are mostly attributed to the invasion and metastasis. It was reported that lymph node metastasis which constituted more than 50% was the foremost section among them, whereas peritoneum metastasis presented 5%‐20%.^4^, ^5^ Hence, the molecular mechanism underlying the progression of GC is necessary to be explored, which may provide a basis for novel therapeutic targets.

RETRACTED

MicroRNAs (miRNAs) are a class of small non‐coding RNAs consisting of 20‐24 nucleotides which can negatively regulate downstream target gene expression.^6^, ^7^ It is well known that miRNAs ectopically expressed in diverse cancers and act as tumour suppressors or oncogenes.^8^, ^9^, ^10^ So, miRNA therapeutics broad a new era for the management of cancer.^11^ MiR‐664a‐3p, located in the intron of RAB3GAP2, has been reported to aberrantly express in various malignancies, including cervical cancer, osteosarcoma, breast cancer and T‐cell acute lymphoblastic leukaemia.^12^, ^13^, ^14^, ^15^ However, the precise role and mechanism of miR‐664a‐3p in gastric cancer have not been elucidated. Our study demonstrated that miR‐664a‐3p was markedly upregulated in GC tissues compared to normal samples, suggesting that miR‐664a‐3p may act as a oncogene in GC.

Mps One Binder Kinase Activator (MOB)1A is one of the most core components of the Hippo pathway.^16^ It has been reported that MOB1A was involved in certain biological behaviours in many types of tumour, such as proliferation, invasion and migration.^17^, ^18^ The decreased expression of hMOB1 mRNA might be the early phase phenomenon for tumour invasion in NSCLC.^19^ Previous study investigated that MOB1A could exert roles as a tumour suppressor through regulating downstream molecular of the Hippo pathway by utilizing kDKO mice.^20^, ^21^ In our study, we discovered that MOB1A is a direct target of miR‐664a‐3p and plays a vital role in GC.

It has been acknowledged that transcription factors could play significant roles in miRNA expression regulation.^22^ Thus, the potential upstream regulator of miR‐664a‐3p required to be explored. Bioinformatic analysis and experimental confirmation indicated that a Foxp3‐binding region presented in the promoter of the miR‐664 gene. Forkhead box protein 3 (Foxp3) is a member of the forkhead/winged helix family of transcription factors.^23^ However, the functions of Foxp3 on different cancer are controversial.^24^, ^25^, ^26^ Our previous research found that ectopic tumoral Foxp3 can promote gastric cancer proliferation, migration and invasion.^27^ Therefore, it is necessary to verify whether Foxp3 is involved in miR‐664a‐3p/MOB1A axis.

RETRACTED

## 2 MATERIALS AND METHODS

### 2.1 Tissue samples and cell lines

The specimens were surgically obtained from the Department of General Surgery, First Affiliated Hospital of Nanjing Medical University. No radiotherapy or chemotherapy was conducted before surgery and patients or their relatives signed informed consents. This study was approved by the First Affiliated Hospital of Nanjing Medical University Ethics Committee. Human GC cell lines, AGS, MGC803, BGC823, HGC27, SGC7901, MKN45 and non‐malignant gastric epithelium cell line GES‐1 were purchased from the Cell Center of Shanghai Institutes for Biological Sciences. All cell lines were cultured in RPMI‐1640 medium (Gibico, Carlsbad, CA, USA) supplemented with 10% foetal bovine serum (Gibico) and 1% penicillin/streptomycin (Gibico) at 37°C in a humidified cell chamber with an atmosphere of 5% CO_2_.

### 2.2 RNA extraction and PCR

Total RNA was extracted from GC tissues and cells by using TRIzol reagent (Invitrogen, Carlsbad, CA, USA) according to the manufacturer's protocols. U6 and β‐actin were used as endogenous controls to normalize miRNA and mRNA, respectively. The relative expression level was quantified using the $2^{-\Delta \Delta C_{\text{T}}}$ method. PCR for each sample was performed in triplicate. All primers (Realgene, Nanjing, China) used in our study were as follow: hsa‐miR‐664a‐3p: forward, 5′‐ACACTCCAGCTGGGTATTCATTTATCCCCAGCC‐3′; universal, 5′‐GCGAGCACA GAATTAATACGAC‐3′; U6 forward, 5′‐CTCGCTTCGGCAGCACA‐3′; reverse, 5′‐AACGCT TCACGAATTTGCGT‐3′; MOB1A forward, 5‐TTGTAAGTGGGTCTGAATAGC; reverse, 5‐GGTGAAAGGTAATGGCATCT; β‐actin forward, 5′‐GCATCGTCACCAACTGGGAC‐3′; reverse, 5′‐ACCTGGCCGTCAGGCAGCTC‐3′; Foxp3 forward, 5′‐TACTTCAAGTTCCAC AACATGCGACC‐3′; reverse, 5′‐CGCACAAAGCACTTGTGCAGACTCAG‐3′.

### 2.3 Colony formation assay

Each group of stable transfected GC cells was plated in six‐well plates (500 cells/well) and cultured in RMPI‐1640 medium for 3 weeks. The colonies were stained with crystal violet after washing away with PBS.

### 2.4 5‐Ethynyl‐2′‐deoxyuridine (EdU) assay

Cell proliferation was measured using the EdU assay kit (RiboBio, Guangzhou, China). Firstly, cells were seeded into 96‐well plates (2 × 10^4^ cells/well) and cultured with complete medium for 24 hours before the addition of EdU (50 μmol/L). Then, cells were incubated for 2 hours at 37°C, fixed in 4% formaldehyde for 30 minutes and permeabilized with 0.5% TritonX‐100 for 10 minutes at room temperature. After washing with PBS, 1×ApolloR reaction cocktail (400 μL) was added to react with the EdU for 30 minutes. Next, Hoechest33342 (400 μL) was added for 30 minutes to visualize the nuclei. Finally, images of cells were captured under a microscope.

RETRACTED

### 2.5 Invasion and migration assay

We used 24‐well BioCoat Matrigel Invasion Chambers (BD Biosciences, Franklin, New Jersey, USA) to evaluate migratory and invasive abilities of GC cells. 3 × 10^4^/well cells were suspended in 200 μL serum‐free medium and were seeded into the upper chamber containing an uncoated or matrigel‐coated membrane, and then complete medium (700 μL) was added into lower chamber. 0.1% crystal violet was used to stain the cells that invaded or migrated to the low membrane after 24‐hour incubation at 37°C in a humidified 5% CO_2_ incubator. The experiments were performed in triplicates.

### 2.6 Immunohistochemistry

All samples were fixed in 4% formaldehyde solution and embedded in paraffin. Then, paraffin‐embedded sections were de‐waxed in xylene and were rehydrated in graded alcohols. The sections were then incubated with primary antibodies anti‐MOB1A followed by secondary antibody conjugated with HRP. Subsequently, detection was conducted by 3,3′‐diaminobenzidine and haematoxylin. We selected three randomly fields for examination.

### 2.7 Western blotting

The proteins were extracted from GC tissues and cells according to manufacturer's instruction. The concentration of proteins was determined by BCA. Then, the proteins were separated by 10% SDS‐PAGE and transferred onto PVDF membranes. Following, membranes were blocked with 5% non‐fat milk at room temperature for 2 hours, and incubated with specific primary antibodies overnight at 4°C, and then incubated with HRP‐conjugated secondary antibodies at room temperature for 2 hours. Finally, membranes were detected by Enhanced Chemiluminescence Detection Kit after washing with TBST buffer three times.

### 2.8 Dual luciferase reporter assay

The 3ʹ‐UTR sequences of MOB1A containing mutant (mut) or wild‐type (wt) miR‐664a‐3p binding sites were constructed by Genscript (Nanjing, China) and cloned into pGL‐3 luciferase reporter vector. Cells were co‐transfected with either the pGL3‐WT‐MOB1A or the pGL3‐MUT‐MOB1A 3′‐UTR reporter plasmids together with miR‐664a‐3p mimic or NC using Lipofectamine 3000 (Invitrogen) after incubation for 24 hours in 24‐well plate. In a next experiment, wild‐type or mutated Foxp3‐binding site reporter was constructed by GeneCopoeia (Nanjing, China) and was co‐transfected together with Foxp3 expression vector into HEK293 cells. Firefly and Renilla luciferase activity was assessed by the Dual‐Luciferase Assay System (Promega, Madison, WI, USA). The relative expression of firefly luciferase activity was normalized to Renilla luciferase activity. The experiment was performed in triplicate.

RETRACTED

### 2.9 Chromatin immunoprecipitation assay

ChIP assay was performed using an EZ‐Magna ChIP kit (Millipore, Darmstadt, Germany) according to the manufacturer's instructions. Briefly, 2 × 10^6^ cells were cross‐linked with 1% formaldehyde for 15 minutes at room temperature and then quenched by adding 0.125 mol/L glycine. The cells were rinsed twice with PBS and collected after 5‐minute centrifugation at 800 *g* at 4°C. The samples were resuspended in 1% SDS lysis buffer, and the chromatin was sheared into 400‐bp fragment using an Ultrasonic Cell Disruptor (Covaris, Waltham, MA, USA). Foxp3 was immunoprecipitated from the supernatant using an anti‐Foxp3 antibody (normal rabbit IgG antibodies were used as negative controls) at 4°C with rotation for 16 hours. The complexes collected by magnetic beads were rinsed and eluted with 1% SDS and 0.1 mol/L NaHCO3, and DNA was purified on spin columns. Promoter binding was tested by PCR with SYBR Green Master Mix (Takara, Beijing, Japan). Enrichments were presented as percentage of the input.

### 2.10 Animal experiment

In this study, all the animal experiments were approved by Nanjing Medical University Ethics Committee. Four‐week‐old female nude mice (BALB/c nude mice) were purchased from the Department of Laboratory Animal Center of Nanjing Medical University. Stably transfected cells (2 × 10^6^ cells) resuspended in 100 μL PBS were injected into tail vein of mice, respectively. After 5 weeks, we observed the occurence of distance metastases using IVIS Imaging system (Caliper life Sciences, Hopkinton, MA, USA).

### 2.11 Statistical analysis

All data are presented as mean ± SD of at least three independent experiments. Differences between two groups were analysed by Student's *t* test. The association of miR‐664a‐3p or MOB1A with clinicopathologic features was analysed by the *χ^2^* test. The linear correlation coefficient (Pearson *r*) was utilized to assess the correlation between miR‐664a‐3p and MOB1A levels in the matched GC tissues. Survival analysis of mice was assessed by Kaplan‐Meier plots. All of the data were analysed using SPSS19.0 software (SPSS, New Orchard Road, Armonk, New York, USA) and were considered to be statistically significant when *P* values were <0.05.

## 3 RESULTS

### 3.1 miR‐664a‐3p is upregulated in GC tissues and cells and promotes GC cell proliferation

We found that miR‐664a‐3p expression was significantly upregulated in GC samples compared to normal cases (Figure 1A). We further examined miR‐664a‐3p expression in six GC cell lines and a normal epithelial cell line (GES‐1). It was shown that miR‐664a‐3p was increased in GC cell lines (AGS, MGC803, BGC823, HGC27, MKN45, SGC7901) compared with GES‐1 (Figure 1B). SGC7901 and HGC27 were chosen for further investigation. We also found that expression of miR‐664a‐3p was higher in metastasis group compared to non‐metastasis group (Figure 1C). As shown in Table 1, in tumour size larger than 3 cm and lymph node metastasis group, the level of miR‐664a‐3p was markedly upregulated. Moreover, GC patients with high expression of miR‐664a‐3p had significantly shorter overall survival than those with the low expression of miR‐664a‐3p by the analysis of Kaplan‐Meier survival curve (*P* < 0.05) (Figure 1D). Further Cox multivariate survival analysis revealed that high miR‐664a‐3p expression was an independent prognostic factors for poor survival of GC patients (hazard ratio [HR] = 2.31, 95% confidence interval [CI] 1.98‐5.57, *P* = 0.013) (Table 2). To explore the role of miR‐664a‐3p in GC, we transfected miR‐664a‐3p mimics, negative control and inhibitor lentivirus in SGC7901 and HGC27, respectively. Compared with the, respectively, negative control group, miR‐664a‐3p expression levels were notably elevated in mimic group and reduced in inhibitor group (Figure 1E,F). After that, we explore the biological functions of miR‐664a‐3p in GC. In mimic group, the proliferation rate was increased in SGC 7901 and HGC27 while decreased in inhibitor group compared to that of the relative control group (Figure 1G). Then, EdU incorporation assay and colony formation assay were used for further evaluation of the effect of miR‐664a‐3p on proliferation (Figure 1H,I). The results showed that overexpression of miR‐664a‐3p enhanced colony formation ability while miR‐664a‐3p knockdown showed the opposite effects (Figure 1J). As shown in Figure 1J, the number of GC cells incorporation EdU in mimic group was increased compared with that in control group, while that was decreased in inhibitor group (Figure 1K).

RETRACTED

**Figure 1:** Relative expression of miR‐664a‐3p in GC tissues and cell lines. A, The relative expression of miR‐664a‐3p in 58 pairs of human GC tissues and normal tissues. B, The relative expression of miR‐664a‐3p in GC cells and GES‐1. C, The expression of miR‐664a‐3p in metastasis group compared to non‐metastasis group. D,E, The relative expression of miR‐664a‐3p in cells after tansfection of miR‐664a‐3p mimic, NC and inhibitor lentivirous, respectively, in SGC7901 and HGC27. F, CCK‐8 was used to determine the proliferation of GC cells transfected with miR‐664a‐3p mimic and inhibitor lentivirus in SGC7901 and HGC27. G,H, Representative profiles of EdU assay and colony formation assay in miR‐664a‐3p mimic and inhibitor groups in SGC7901 and HGC27. I,J, The number of colony formation and rate of EdU positive cells were counted in miR‐664a‐3p mimic and inhibitor groups. *P < 0.05, **P < 0.01, ***P < 0.001. The data expressed as the mean ± SD

**Table 1:** Expression of miRNA‐664a‐3p expression and MOB1A in human gastric cancer according to patients’ clinicopathological characteristics

Characteristics	Number	miR‐664a‐3p expression		*P* values	MOB1A expression		*P* values
		High group	Low group		High group	Low group	
Age (yr)							
<60	19	10	9	0.779	11	8	0.401
≥60	39	19	20		18	21	
Gender							
Male	28	15	13	0.599	11	17	0.115
Female	30	14	16		18	12	
Size(cm)							
<3	28	10	18	0.035*	18	10	0.035*
≥3	30	19	11		11	19	
Histology grade							
Well/Moderately	22	11	13	0.593	12	10	0.583
Poorly	36	18	16		17	19	
Stage							
I/II	34	12	22	0.015*	21	13	0.033*
III/IV	24	17	7		8	16	
N stage							
Present (N1‐N3)	33	21	12	0.033*	11	22	0.004^**^
Absent (N0)	25	8	17		18	7	

* *P* < 0.05 statistically significant difference, **P < 0.01.

**Table 2:** Univariate and multivariate overall survival analysis of prognostic factors for GC patients

Characteristics	Overall survival (n = 58)					
	Univariate analysis			Multivariate analysis		
	HR	95%CI	*P* value	HR	95%CI	*P* value
Age (<60 vs ≥60 yr)	0.89	0.31‐2.54	0.821			
Gender (male vs female)	1.08	0.41‐2.86	0.879			
Tumour size (<3 vs ≥3 cm)	1.64	1.22‐5.73	0.032*	0.57	0.81‐4.23	0.732
Differentiation (well/moderate vs poor)	0.89	0.48‐3.75	0.749			
TNM stage (I‐II vs III‐IV)	4.53	1.94‐6.82	0.003**	3.34	1.14‐4.87	0.024*
Lymph node metastasis (N0 vs N1‐3)	4.01	2.83‐7.97	<0.001***	1.94	1.84‐4.71	0.039*
miR‐664a‐3p expression (High vs Low)	4.75	2.48‐8.95	0.007**	2.31	1.98‐5.57	0.013*

*P < 0.05, **P < 0.01, ***P < 0.001.

### 3.2 miR‐664a‐3p enhances invasion, migration and the EMT processing in GC cells

The wound‐healing assay and transwell assay were performed, and the results illustrated that the overexpression of miR‐664a‐3p in mimic group exerted active effect on GC cell invasion and migration (Figure 2A,B), while the downexpression of miR‐664a‐3p in inhibitor group showed opposite influence (Figure 2C,D). These data indicated that miR‐664a‐3p enhances cell invasion and migration of GC.

**Figure 2:** miR‐664a‐3p facilitates invasion, migration and EMT process in vitro. A,B, Wound‐healing assay was used to determine the migration of GC cells after transfection of miR‐664a‐3p mimic, NC and inhibitor lentivirous, respectively, in SGC7901 and HGC27. C,D, Effects of miR‐664a‐3p alteration on invasion and migration by transwell assay in vitro. E, Effects of miR‐664a‐3p on EMT process analyzed by Gene Set Enrichment Analysis (GSEA). F, The expression of EMT‐associated proteins detected by Western blot when expression of miR‐664a‐3p was altered in SGC7901 and HGC27. G,H, The Immunofluorescence assay of Ecadherin (red) and Vimentin (green) in SGC7901 and HGC27. The nucleus staining with DAPI (blue).*P < 0.05, **P < 0.01, ***P < 0.001. The data expressed as the mean ± SD

To clarify whether miR‐664a‐3p has impact on the EMT processing of GC cells, we first analysed that by Gene Set Enrichment Analysis (GSEA) and it showed that miR‐664a‐3p expression was positively correlated with EMT‐associated gene signatures (Figure 2E). Therefore, we evaluated the expression of EMT markers by using immunofluorescence analysis after transfection. The results revealed that the level of E‐cadherin (epithelial marker) was descended while Vimentin (mesenchymal marker) was rose in the mimic group, whereas it was contrast in the inhibitor group (Figure 2G,H). Moreover, Western blot analysis indicated that upregulation of miR‐664a‐3p expression increased the level of the epithelial marker (E‐cadherin) and attenuated the levels of the mesenchymal marker (N‐cadherin, Vimentin) and transcription factors (Slug, Snail). While downregulation of miR‐664a‐3p expression showed opposite (Figure 2F). These results demonstrated that miR‐664a‐3p might play a critical role on EMT progression thereby contributing to the invasion and migration of GC cells in vitro.

RETRACTED

### 3.3 MOB1A is a direct target of miR‐664a‐3p and downregulated in GC tissues and cells

We utilized bioinformatics miRNA target prediction programs (Targetscan, starBase, PicTar and miRanda) to search for potential miR‐664a‐3p target genes. MOB1A was selected as a candidate since it has a latent miR‐664a‐3p‐binding site in its 3′‐UTR.

To assess the association between miR‐664a‐3p and MOB1A expression in GC tissues, we performed qRT‐PCR to analyse MOB1A expression in 58 pairs of GC tissue and matched adjacent non‐cancerous tissue samples. The outcomes proclaimed that the expression of MOB1A was downregulated in GC tissues (Figure 3A). We further confirmed the downexpression of MOB1A in six pairs GC tissues via Western blotting and immunohistochemistry, representative results were shown in Figure 3B,C. Also, we concluded that MOB1A expression level was lower in GC cell lines than that in GES‐1 (Figure 3D). Furthermore, high expression of MOB1A contributed to better prognosis on the public database Kaplan‐Meier Plotter (http://kmplot.com/analysis/) (Figure 3E). Moreover, we obtained that expression of miR‐664a‐3p was negatively correlated with that of MOB1A (Figure 3F). We also evaluated the relevant between the MOB1A expression with patients’ clinicopathological characteristics (Table 1).

RETRACTED

**Figure 3:** MOB1A is a direct target of miR‐664a‐3p and downregulated in GC tissues and cells. A, The relative expression of miR‐664a‐3p in 58 pairs of GC tissues. B, The expression of MOB1A was detected in six pairs of GC samples by Western blot. C, Representative IHC staining of MOB1A in six pairs of GC and normal specimens. D, The relative expression of MOB1A in GC cells compared to GES‐1. E, The survival analysis of MOB1A on the Kaplan‐Meier Plotter. F, Negative relation between of miR‐664a‐3p and MOB1A in GC tissues. G, Luciferase reporter assay was conducted to confirm that miR‐664a‐3p directly binded to the 3′‐UTR region of MOB1A. H, The relative expression of MOB1A after transfection of miR‐664a‐3p mimic, NC and inhibitor lentivirous by qRT‐PCR. I, Relative luciferase activity was analyzed in GC cells co‐transfcted miR‐664a‐3pmimics or NC with pGL3‐MOB1A‐WT or pGL3‐MOB1A‐MUT, respectively. J, Western blot was ultilized to determine the expression of MOB1A when miR‐664a‐3p expression was altered in GC cells

We further verified whether miR‐664a‐3p could directly target the 3′‐UTR of MOB1A mRNA by dual‐luciferase reporter assay. Wild‐type (WT) and mutant‐type (MUT) MOB1A 3′UTR sequences were subcloned into the pGL3 luciferase reporter vector. We noticed that the co‐transfection with miR‐664a‐3p mimic and pGL3‐MOB1A‐WT 3′UTR led to declined luciferase activity compared to that in control group (pGL3‐MOB1A‐MUT 3′UTR) (Figure 3G,H). We observed that increased expression of miR‐664a‐3p could obviously depress the mRNA and protein level of MOB1A, while knockdown expression of miR‐664a‐3p displayed reverse effect (Figure 3I,J). Taken together, our results suggested that MOB1A was a direct target of miR‐664a‐3p and was frequently downregulated in GC tissues and cells.

### 3.4 MOB1A reverses the effects of miR‐664a‐3p on GC cells

To further verify whether the effects of miR‐664a‐3p on invasion and migration in GC cells were mediated by ectopic expression of MOB1A, we overexpressed MOB1A by constructing lentiviral vector (Lv‐MOB1A) and inhibited by sh‐MOB1A. Our results showed that co‐transfection of Lv‐MOB1A in miR‐664a‐3p mimic cells reversed the promotional function of miR‐664a‐3p in EdU assay and colon formation assay (Figure 4A,B). Then, we knocked down the level of MOB1A in miR‐664a‐3p inhibitor cells, as expected, we concluded that decline of MOB1A eliminated the impact of miR‐664a‐3p inhibition on GC cells migration (Figure 4A,B). The numbers of colon formation were counted in Figure 4C and the rates of EdU‐positive cells in different groups were shown in Figure 4D. We obtained similar results via wound‐healing assay and transwell assay (Figure 4E‐H). The numbers of invasive and migratory cells were counted (Figure 4I,J).

RETRACTED

**Figure 4:** MOB1A restores the effects of miR‐664a‐3p on GC cells. A,B, Co‐transfection of Lv‐MOB1A in miR‐ 664a‐3p mimic cells reversed the promotional function of miR‐664a‐3p in EdU assay and colon formation assay in SGC7901 and HGC27. C,D, The number of colony formation and rate of EdU positive cells were counted in different groups. E,F, Wound‐healing assay was used to verify the rescuement effects of MOB1A on migration of GC cells. G,H, MOB1A eliminated the roles of miR‐664a‐3p on invasion and migration in SGC7901 and HGC27 using transwell assay. I,J, The cells counts of transwell assay in SGC7901 and HGC27. K,L, The expression of EMT‐associated proteins was detected when Lv‐MOB1A or sh‐MOB1A tranfected into miR‐664a‐3p mimic or inhibitor group in vitro. M,N, The immunofluorescence assay of E‐cadherin (red) and Vimentin (green) in SGC7901 and HGC27 after co‐transfection. The nucleus staining with DAPI (blue). *P < 0.05, **P < 0.01, ***P < 0.001. The data expressed as the mean ± SD

Subsequently, we applied immunoflurosence and Western blotting analysis to confirm whether miR‐664a‐3p accelerated the EMT progression of GC cells by targeting MOB1A. The fluorescence intensity of E‐cadherin was strengthened when stable transfected Lv‐MOB1A in miR‐664a‐3p mimic cells, while was weakened after transfection of sh‐MOB1A in miR‐664a‐3p inhibition cells. The fluorescence intensity of Vimentin showed opponent results (Figure 4M,N). Similarly, in Western blot assay, E‐cadherin expression was significantly increased when stable transfected Lv‐MOB1A in miR‐664a‐3p mimic cells, while decreased after transfection of sh‐MOB1A in miR‐664a‐3p inhibitior cells. Other related proteins (N‐cadherin, Vimentin, Snail, Slug) levels appeared opposite events (Figure 4K,l). The above results provided additional evidence that miR‐664a‐3p magnified GC process by targeting MOB1A directly in vitro.

### 3.5 miR‐664a‐3p contributes to tumour progression and metastasis in vivo

We performed xenograft assays to further validate the role of miR‐664a‐3p on tumour progression. SGC7901 and HGC27 cells transfected as described above were injected into the flanks of nude mice. As shown in Figure 5A‐C, the tumour volume and weight in miR‐664a‐3p mimic group were increased, while those were decreased in miR‐664a‐3p inhibitor group compared with those in miR‐NC group. Ki67 staining assay was used to further verify that miR‐664a‐3p promoted tumorigenicity. The Ki67‐positive ratio was higher in miR‐664a‐3p mimic group, while the opposite trend was shown in miR‐664a‐3p inhibitor group compared with that in miR‐NC group (Figure 5D,E). Furthermore, Western blot assay of tumour in mice indicated significant downregulation of MOB1A expression in miR‐664a‐3p mimic group, which was contrast in miR‐664a‐3p inhibitor group (Figure 5F). To validate the function of miR‐664a‐3p on tumour metastasis in vivo, stable transfected cells were injected into tail vein of BALB/c nude mice separately. After 6 weeks, we found a significant promotion on lung metastasis in miR‐664a‐3p mimic group compared to that in miR‐NC group. We also found a alleviation on lung metastasis in miR‐664a‐3p inhibitior group compared to that in miR‐NC group (Figure 5G). After that, mice were euthanized and then lung tissues were examined by H&E staining, which showed consistently results (Figure 5H). Collectively, these results demonstrated that miR‐664a‐3p could facilitate tumour progression and metastasis in vivo.

RETRACTED

**Figure 5:** miR‐664a‐3p promotes metastasis of GC in vivo. A, photographs of tumors obtained from mice in miR 664a‐3p mimic and inhibitor groups. B,C, tumor volume and weight were calculated in miR‐664a‐3p mimic and inhibitor groups in SGC7901 and HGC27. D,E, Ki67 staining assay was used to further verify that miR‐664a‐3p promoted tumorigenicity. The Ki67 positive ratio was higher in miR‐664a‐3p mimic group, while the opposite trend was shown in miR‐664a‐3p inhibitor group compared with that in miR‐NC group. F, Western blot assay of tumor in mice indicated significant downregulation of MOB1A expression in miR‐664a‐3p mimic group, which was contrast in miR‐664a‐3p inhibitor group. *P < 0.05, **P < 0.01, ***P < 0.001. The data expressed as the mean ± SD. G, Representative photographs of tumors were taken by the IVIS Imaging System in different groups. H, Representative H&E‐stained sections of lung from mice in different groups.

### 3.6 Elevated expression of miR‐664a‐3p promotes GC progression by targeting MOB1A through inactivation of the hippo pathway

MOB1A is a important component of the Hippo pathway, which has been reported to be involved in tumour metastasis.^28^, ^29^ LATS1/2 are phosphorylated and activated by upstream molecules MST1/2, while MOB1A could associated with LATS1/2 to manifest its phosphorylation and potentiate its catalytic activity.^30^ Accumulating evidence demonstrated that activated LATS1/2 directly stimulate phosphorylation of the key transcriptional coactivators YAP and TAZ, which make YAP and TAZ trap within the cytoplasm.^31^ Dephosphorylation of YAP and TAZ duing to repression of phosphorylated LATS1/2 leads to the enrichment of YAP and TAZ in nucleus, which in turn causing negative impact on the downstream Hippo cascades.^32^

RETRACTED

In our study, we verified that YAP and TAZ gathered more in nucleus due to the decline of MOB1A when miR‐664a‐3p was increased. In miR‐664a‐3p mimic cells, p‐LATS2, p‐YAP and p‐TAZ was reduced as a result of downexpression of MOB1A while we drawn a counter conclusion in miR‐664a‐3p inhibitor cells (Figure 6A,B). Subsequently, the expression of YAP and TAZ in nucleus was increased when miR‐664a‐3p was overexpressed both in SGC7901 and in HGC27 (Figure 6C,D). Immunofluorescence assay displayed analogous tendency (Figure 6E,F). Additionally, we confirmed that ectopic expression of MOB1A could restore the effect of miR‐664a‐3p. The expression of p‐LATS2, p‐YAP and p‐TAZ was restored after co‐transfection in SGC7901 and HGC27, respectively (Figure 6A,B). Simultaneously, the accumulation of YAP and TAZ in nucleus was altered (Figure 6C,D), and the fluorescence intensity of YAP and TAZ exhibited correspondingly result (Figure 6E,F). As expected, these findings were consistent with our postulation that elevated expression of miR‐664a‐3p promotes GC metastasis by targeting MOB1A through inactivation of the Hippo pathway.

**Figure 6:** miR‐664a‐3p plays a role in GC cells by directly targeting MOB1A through inactivation of the Hippo pathway. A,B, The alteration of downstream moleculars of the Hippo pathway detected by Western blot. C,D, Elevation of miR‐664a‐3p expression contributed to the trap of YAP and TAZ in nucleus. E,F, YAP and TAZ was accumulated in nucleus in SGC7901 and HGC27, respectively, by immunofluorescence analysis due to increase of miR‐664a‐3p expression and MOB1A could rescue the effects

### 3.7 Foxp3 activates miR‐664a‐3p expression

Our previous research found that ectopic tumoral Foxp3 can promote gastric cancer proliferation, migration and invasion. In present study, we found that Foxp3 mRNA level was significantly upregulated in GC tissues (Figure 7A) and cell lines (Figure 7B). The public database Kaplan‐Meier Plotter (http://kmplot.com/analysis/) displayed that high expression of Foxp3 in GC samples was associated with markedly decreased five‐year overall survival (Figure 7C). Applying the JASPAR database (http://jaspar.genereg.net/) and the UCSC genome browser tool (http://genome.ucsc.edu/index.html), we speculated that Foxp3 might bind to miR‐664a‐3p promoter and activate its expression (Figure 7D). We constructed the Foxp3‐binding site reporter and transfected into HEK293 cells and found that the Foxp3‐binding site‐WT reporter had higher luciferase activity compared to the mutant reporter (Figure 7E). Correspondingly, the ChIP results illustrated that Foxp3 binds to the putative binding site upstream of miR‐664 (Figure 7F). The expression level of miR‐664a‐3p was increased when Foxp3 was upregulated while decreased with the decline of Foxp3 level in SGC7901 and HGC27 (Figure 7G,H). Overexpression of Foxp3 in GC cells led to reduced MOB1A expression and the opposite influence occurred in the Foxp3 downregulated group (Figure 7I,J). Accordingly, these data indicated that Foxp3 mediated miR‐664a‐3p promotion of GC progression by targeting MOB1A through the inactivation of the Hippo pathway.

RETRACTED

**Figure 7:** Foxp3 actives miR‐664a‐3p expression. A, The expression of Foxp3 in 58 pairs of GC specimens. B, The expression of Foxp3 in GC cells compared to GES‐1. C, The survival analysis of Foxp3 on the Kaplan‐Meier Plotter. D, Bioinformatic analysis indicated that Foxp3 might bind to miR‐664a‐3p promoter. E, Relative luciferase activity was analyzed in HEK293 cell. F, ChIP assay was performed with control (rat IgG), anti‐Foxp3 antibody to determine Foxp3 occupancy of miR‐664a‐3p promoter. G,H, The relative expression of miR‐664a‐3p altered when transfected Lv‐Foxp3, Pex3, and sh‐Foxp3 in SGC7901 and HGC27. Pex3 was control vector. I,J, qRT‐PCR was used to detected the relative expression of MOB1A when the level of Foxp3 was altered

## 4 DISCUSSION

Emerging evidence showed that miRNAs could exert different effects on the progression of cancers depending on targeting downstream genes. MiRNAs downregulate gene expression by binding to the 3′‐untranslated regions of downstream target gene, resulting in inhibition of translation or mRNA degradation.^8^, ^33^ MOB1 (encoded by MOB1A and MOB1B in human) is an important component of the Hippo pathway, which was considered to influence biological functions in many tumours.^17^, ^34^, ^35^, ^36^ It has been reported that MOB1 directly binds to LATS1 and LATS2, and additionally to two related kinases, NDR1and NDR2 via a specialized MOB1‐binding domain.^37^ Dephosphorylation of YAP and TAZ duing to repression of phosphorylated LATS1/2 leads to the enrichment of YAP and TAZ in nucleus, which in turn causing negative impact on the downstream Hippo cascades.^32^, ^38^

Foxp3 is a member of the forkhead/winged helix family of transcription factors. It has been reported to play various roles in different cancer types.^39^, ^40^, ^41^ Other study indicated that transcription factor could regulate expression of miRNAs to play critical roles in various types of cancer.^42^, ^43^

To the best of our knowledge, our study firstly demonstrated that miR‐664a‐3p was frequently upregulated in GC tissues and cell lines and acted as a oncogene by targeting downstream MOB1A through inactivation of the Hippo pathway. However, the more concrete downstream molecular alteration of the Hippo pathway and the exact mechanism of phosphorylation of YAP and TAZ affected by miR‐664a‐3p need further investigation. Overall, we expect that our findings for Foxp3/miR‐664a‐3p/MOB1A/Hippo pathway axis will furnish certain promising strategies for the therapy of GC.

RETRACTED

## CONFLICT OF INTEREST

The authors declare that they have no conflict of interest.
